# Efficacy of Bevacizumab and Gemcitabine in Combination with Cisplatin in the Treatment of Esophageal Cancer and the Effect on the Incidence of Adverse Reactions

**DOI:** 10.1155/2022/2317181

**Published:** 2022-04-18

**Authors:** Jiangfeng Wang, Qiang Zhao, Lei Cai, Jianqiang Li, Sheng Chen

**Affiliations:** Department of Thoracic Surgery, Institute of Cancer Research and Basic Medical Sciences of Chinese Academy of Sciences, Cancer Hospital of University of Chinese Academy of Sciences, Zhejiang Cancer Hospital, No. 1 Banshan East Road, Gongshu District, Hangzhou, 310022, China

## Abstract

**Objective:**

To evaluate the efficacy of bevacizumab and gemcitabine in combination with cisplatin in the treatment of esophageal cancer and the effect on the incidence of adverse reactions.

**Methods:**

A total of 100 esophageal cancer patients admitted to our hospital from March 2019 to March 2021 were identified as research subjects and randomized into the control group and the study group, with 50 cases in each group. The control group was treated with gemcitabine combined with cisplatin, and the study group was treated with the triple therapy of bevacizumab, gemcitabine, and cisplatin. The treatment efficiency and the incidence of adverse reactions were compared between the two groups of patients.

**Results:**

The total treatment efficiency in the study group was 86%, which was significantly higher than that of 66% in the control group (*P* < 0.05). After treatment, the levels of vascular endothelial growth factor (VEGF), Cyfra21-1, and C-met were reduced in both groups, with significantly lower levels in the study group than in the control group (*P* < 0.05). The incidence of all CTCAE, ototoxicity, and nephrotoxicity was comparable between the two groups (*P* > 0.05). The survival rates of patients in the study group were 88% and 54% at 1 and 2 years after treatment, which were significantly higher than that of 68% and 32% in the control group (*P* < 0.05).

**Conclusion:**

The clinical efficiency of bevacizumab and gemcitabine combined with cisplatin in the treatment of esophageal cancer is remarkable, which improves the survival of patients, and is worthy of clinical promotion and application.

## 1. Introduction

Esophageal cancer is a malignant tumor that occurs in the epithelial tissue of the esophagus, with a growing incidence that accounts for about 2% of all malignancies [1]. The incidence of esophageal cancer varies widely from region to region, and China is a country with a high morbidity and mortality rate of esophageal cancer [2]. The clinical staging of esophageal cancer, including early, middle, and advanced stages, is related to chronic stimulation of nitrosamines, inflammation, trauma, and genetic factors. In addition, smoking and drinking are also common causes of esophageal cancer, for which treatment includes surgery, chemotherapy, and drug therapy [3–5]. Bevacizumab is a monoclonal antibody that inhibits vascular endothelial growth factors and affects vascular permeability, proliferation, and endothelial cell migration and survival to suppress tumor angiogenesis, growth, and metastasis [6, 7]. Gemcitabine combined with cisplatin is a commonly used chemotherapy regimen to improve immunity through the reinfusion of immune cells, to further inhibit and kill residual tumor cells for the control of disease progression, and the prolongation of patient's survival [8, 9]. It has been demonstrated [10] that the combination of bevacizumab with chemotherapeutic drugs enhances antitumor efficacy, which may be broadly related to the ability of bevacizumab to reduce tissue interstitial pressure within the tumor and enhance the penetration of chemotherapeutic drugs within the tumor. This study was conducted to evaluate the efficiency of bevacizumab and gemcitabine in combination with cisplatin in the treatment of esophageal cancer and the effect on the incidence of adverse reactions, which is reported as follows.

## 2. Materials and Methods

### 2.1. General Data

One hundred cases of esophageal cancer patients admitted to our hospital from March 2019 to March 2021 were identified as the study subjects and randomized into the control group and the study group, with 50 cases in each group.

### 2.2. Inclusion Criteria and Exclusion Criteria

Inclusion criteria are as follows: (1) patients who were diagnosed with esophageal cancer after examination; (2) patients with no use of other antitumor drugs for 1 month before treatment; (3) patients with complete clinical data; and (4) the study was approved by the hospital ethics committee, and the patients and their families were informed of the purpose and process of this experimental study and signed the informed consent form.

Exclusion criteria are as follows: (1) patients with serious infectious diseases; (2) patients with psychiatric diseases; (3) patients with esophageal cancer compressing the airway; and (4) patients with withdrawal from the study.

### 2.3. Methods

The control group was treated with gemcitabine combined with cisplatin. 1000 mg/m^2^ gemcitabine (manufacturer: Qilu Pharmaceutical (Hainan) Co., Ltd.; state drug quantification: H20113286; specification: 1.0 g) was added to 250 ml of 0.9% sodium chloride injection for 8 days of intravenous infusion. 20 mg/m^2^ cisplatin (manufacturer: Qilu Pharmaceutical Co., Ltd.; state drug quantification: H37021356; specification: 30 mg) was dissolved in 250 ml of 5% dextrose injection for 8 days of intravenous drip. One treatment cycle spanned 3 weeks, and patients were treated for 4 consecutive cycles.

The study group was treated with bevacizumab (manufacturer: Xinda Biopharmaceutical (Suzhou) Co., Ltd; state drug administration: S20200013; specification: 4 ml: 100 mg) on the basis of the control group by intravenous infusion of 7.5 mg/kg, once/day, on the first day of each treatment cycle. One treatment cycle spanned 3 weeks, and patients were treated for 4 consecutive cycles.

### 2.4. Observation Indexes and Evaluation Criteria

(1) According to the criteria of Response Evaluation Criteria in Solid Tumors (RECIST) 1.1 [11], the treatment efficiency was classified as complete remission (CR), partial remission (PR), stable disease (SD), and disease progression (PD). The treatment efficiency = CR + PR. (2) 5 ml of peripheral venous blood was collected from patients and centrifuged at 2000 r/min for 20 min, and the supernatant was collected and stored frozen at -80°C. Serum vascular endothelial growth factor (VEGF) levels, serum Cyfra21-1, and C-met levels were determined before and after treatment in both groups using enzyme-linked immunosorbent assay (ELISA). (3) Patients were followed up for 2 years after treatment, and the survival rates of patients in both groups were recorded at 1 year and 2 years after treatment. (4) The patients were evaluated for all toxic reactions according to the criteria for assessing toxic reactions of anticancer drugs established by common adverse event evaluation criteria (CTCAE) version 5.0

### 2.5. Statistical Analyses

The data in this study were processed using the SPSS 20.0, and GraphPad Prism 7 (GraphPad Software, San Diego, USA) was used for image rendering. The count data were expressed by (*n* (%)) using the chi-square test, and the measurement data were expressed by (−*x* ± *s*) using the t-test. *P* < 0.05 was considered statistically significant.

## 3. Results

### 3.1. Comparison of Baseline Data

The two groups had no statistical difference in the comparison of baseline data (*P* > 0.05), as shown in Table 1.

### 3.2. Comparison of Clinical Efficiency

The total treatment efficiency in the study group is 86%, which was significantly higher than that of 66% in the control group (*P* < 0.05), as shown in Table 2.

### 3.3. Comparison of VEGF Levels

No statistical significant difference in VEGF levels between the two groups before treatment was found (*P* > 0.05). After treatment, VEGF levels decreased in both groups, with significantly lower levels in the study group than in the control group (*P* < 0.05) (see Figure 1 for details).

### 3.4. Comparison of Cyfra21-1 Levels

The difference in Cyfra21-1 levels between the two groups of patients before treatment was not statistically significant (*P* > 0.05). After treatment, Cyfra21-1 levels decreased in both groups, with markedly lower levels in the study group than in the control group (*P* < 0.05) (see Figure 2 for details).

### 3.5. Comparison of C-met Levels

There was no statistically significant difference in C-met levels between the two groups of patients before treatment (*P* > 0.05). After treatment, the C-met levels decreased in both groups, with markedly lower levels in the study group than in the control group (*P* < 0.05) (see Figure 3 for details).

### 3.6. Comparison of the Incidence of CTCAE

The incidence of all CTCAE, ototoxicity, and nephrotoxicity sre comparable between the two groups (*P* > 0.05), as shown in Table 3 and Table 4.

### 3.7. Comparison of 1-Year and 2-Year Survival Rates after Treatment

The survival rates of patients in the study group at 1 and 2 years after treatment were 88% and 54%, which were significantly higher than those of the control group at 68% and 32% (*P* < 0.05) (see Table 5 and Figure 4).

## 4. Discussion

Esophageal cancer is a common malignant tumor that occurs in the epithelial tissue of the esophagus. China is a high incidence area for esophageal cancer with a high mortality rate, which poses a serious threat to patient's life safety. The occurrence of esophageal cancer is highly related to daily dietary habits, long-term smoking, and drinking. Esophageal cancer has a significant phenomenon of family gathering, with some regions having families with three or more consecutive generations of esophageal cancer cases. Early symptoms of esophageal cancer patients are rather hidden, with manifestations such as foreign body sensation or choking sensation when swallowing food or pain behind the sternum. Patients in the middle and advanced stages usually exhibit dysphagia, with clinical symptoms such as emaciation, fever, hoarseness, choking on water, vomiting blood, and dyspnea as the disease deteriorates [12, 13].

Gemcitabine, a difluorinated nucleoside antimetabolite anticancer agent that disrupts cell replication, has been shown to be effective in a variety of solid tumors by reducing the total amount of deoxynucleotides required for DNA synthesis and prompting DNA breaks and cell death through the hindrance of DNA strand synthesis [14]. Cisplatin is a conventional chemotherapeutic agent that is extensively used in combination chemotherapy for tumors to destroy DNA and inhibit tumor growth [15]. Moreover, cisplatin enhances the denaturation of broken DNA double strands by gemcitabine, which indicates a synergistic effect of the two drugs. A study [16] showed that gemcitabine combined with cisplatin significantly prolonged the patients' survival with high therapeutic efficiency in the treatment of esophageal cancer. Bevacizumab is a recombinant humanized immunoglobulin G1 (IgG1) monoclonal antibody that inhibits vascular endothelial growth factor, affects vascular permeability and proliferation, and involves in the migration and survival of endothelial cells, which serves to inhibit tumor angiogenesis, growth, and metastasis, and accounts for its extensive use in various types of metastatic cancers [17–19]. In this study, the total treatment efficiency in the study group was 86%, which was significantly higher than that of 66% in the control group (*P* < 0.05), indicating a superior treatment efficiency of triple therapy to that of therapy of gemcitabine combined with cisplatin. VEGF is a highly specific provascular endothelial growth factor that increases vascular permeability and promotes extracellular matrix degeneration and the migration, proliferation, and angiogenesis of vascular endothelial cells. As the most potent proangiogenic factor known, vigorous expression of VEGF is observed in tumor patients [20, 21]. In the current study, the VEGF levels were reduced in both groups after treatment, with significantly lower levels in the study group than in the control group (*P* < 0.05), which was similar to the findings of Sadahiro et al. [22], suggesting that bevacizumab and gemcitabine combined with cisplatin for esophageal cancer could reduce VEGF levels and promote apoptosis of cancer cells. Cyfra21-1 is a marker of epithelial cell carcinogenesis that exists in the plasma as an oligomer, which is proteolytically cleaved and enters the circulation upon cell carcinogenesis [23]. C-met, a member of the receptor tyrosine kinase family, is associated with a variety of oncogene products and regulatory proteins. It has been reported that the tumor C-met signaling pathway can be activated by cancer cells, contributing to tumor formation, aggressive growth, and metastasis [24, 25]. In this study, it was shown that bevacizumab and gemcitabine combined with cisplatin treatment reduced Cyfra21-1 and C-met levels to inhibit the viability of esophageal cancer cells, thereby inhibiting the progression of esophageal cancer. Furthermore, the survival rates of patients in the study group were 88% and 54% at 1 and 2 years after treatment, which were significantly higher than that of 68% and 32% in the control group (*P* < 0.05), suggesting that the triple therapy of bevacizumab, gemcitabine, and cisplatin for esophageal cancer could boost the treatment efficiency, enhance the survival rate, and prolong the survival time of patients with esophageal cancer.

In conclusion, the clinical efficiency of bevacizumab and gemcitabine combined with cisplatin in the treatment of esophageal cancer is remarkable, which reduces the incidence of adverse reactions and improves the survival of patients, and is worthy of clinical promotion and application.

## Figures and Tables

**Figure 1:** Comparison of VEGF levels before and after treatment between two groups of patients (−*x* ± *s*). Note: The abscissa indicates the control group, the study group, and the ordinate indicates the value of VEGF level, ng/L. The VEGF levels before and after treatment in the control group were (547.58 ± 68.44) ng/L and (453.21 ± 54.69) ng/L. The VEGF levels before and after treatment in the study group were (541.75 ± 67.20) ng/L and (394.67 ± 50.18) ng/Ll. ^∗^indicates a significant difference in VEGF levels before and after treatment in the control group (*t* = 7.617, *P* < 0.001). ^∗∗^indicates a significant difference in VEGF levels before and after treatment in the study group (*t* = 12.401, *P* < 0.001). ^∗∗∗^indicates that there is a significant difference in the VEGF levels between the control and study groups after treatment (*t* = 5.577, *P* < 0.001).

**Figure 2:** Comparison of Cyfra21-1 levels in the two groups before and after treatment (−*x* ± *s*). Note: The abscissa indicates before and after treatment, and the ordinate indicates Cyfra21-1 level, pg/L. The Cyfra21-1 levels before and after treatment in the control group were (7.39 ± 0.91) pg/L and (3.67 ± 0.45) pg/L, respectively. The Cyfra21-1 levels before and after treatment in the study group were (7.18 ± 0.84) pg/L and (1.85 ± 0.30) pg/L, respectively. ^∗^indicates a significant difference in Cyfra21-1 levels before and after treatment in the control group (*t* = 25.911, *P* < 0.001). ^∗∗^indicates a significant difference in Cyfra21-1 levels before and after treatment in the study group (*t* = 42.254, *P* < 0.001). ^∗∗∗^indicates a significant difference in Cyfra21-1 levels between the study group and the control group after treatment (*t* = 23.795, *P* < 0.001).

**Figure 3:** Comparison of C-met levels in the two groups before and after treatment (−*x* ± *s*). Note: The abscissa indicates before and after treatment, and the ordinate indicates the C-met level, ug/L. The C-met levels before and after treatment in the control group were (12.04 ± 1.26) ug/L and (6.95 ± 0.61) ug/L. The C-met levels before and after treatment in the study group were (11.73 ± 1.22) ug/L and (3.20 ± 0.39) ug/L. ^∗^indicates a significant difference in C-met levels between the study group and the control group after treatment (*t* = 36.624, *P* < 0.001).

**Figure 4:** Overall survival curve.

**Table 1:** Comparison of baseline data between the two groups (*n* (%)).

Indicators	Control group (*n* = 50)	Study group (*n* = 50)	*χ*2/*t*	*P*
Gender			0.040	0.841
Male	24 (48.00)	23 (46.00)		
Female	26 (52.00)	27 (54.00)		
Average age (years)	48.25 ± 11.34	47.64 ± 11.57	0.266	0.791
Drinker at diagnosis	13 (26.00)	12 (24.00)	0.073	0.787
Smoker at diagnosis	16 (32.00)	14 (28.00)	0.191	0.663
Education level				
University	18 (36.00)	20 (40.00)	0.170	0.680
High school	26 (52.00)	25 (50.00)	0.040	0.841
Elementary school	6 (12.00)	5 (10.00)	0.102	0.749
Family history of esophageal cancer				
Yes	12 (24.00)	11 (22.00)	0.057	0.812
No	38 (76.00)	39 (78.00)		

**Table 2:** Compare the clinical efficiency of patients in the two groups (*n* (%)).

Groups	*n*	CR	PR	SD	PD	Total treatment efficiency
Control group	50	14 (28.00)	19 (38.00)	10 (20.00)	7 (14.00)	33 (66.00)
Study group	50	20 (40.00)	23 (46.00)	5 (10.00)	2 (4.00)	43 (86.00)
*X* ^2^						5.483
*P*						<0.05

**Table 3:** The incidence of all grade CTCAE.

Groups	*n*	Grade I	Grade II	Grade III	Grade IV	Grade V	All grade
Control group	50	18	9	4	2	0	33
Study group	50	21	8	5	2	1	38
*χ* ^2^							1.214
*P*							0.271

**Table 4:** The incidence of ototoxicity and nephrotoxicity.

Groups	*n*	Ototoxicity	Nephrotoxicity
Control group	50	7	9
Study group	50	5	11
*χ* ^2^		0.379	0.250
*P*		0.538	0.617

**Table 5:** Comparison of 1-year and 2-year survival rates after treatment between the two groups of patients (*n* (%)).

Groups	*n*	1 year after treatment	2 years after treatment
Control group	50	34 (68.00)	16 (32.00)
Study group	50	44 (88.00)	27 (54.00)
X^2^		5.828	4.937
*P*		<0.05	<0.05

## Data Availability

No data were used to support this study.

## References

[1] Svaton M., Blazek J., Krakorova G. (2021). Prognostic role for CYFRA 21-1 in patients with advanced-stage NSCLC treated with bevacizumab plus chemotherapy. *Anticancer Research: International Journal of Cancer Research and Treatment*.

[2] Leslie K. K., Filiaci V. L., Mallen A. R. (2021). Mutated p53 portends improvement in outcomes when bevacizumab is combined with chemotherapy in advanced/recurrent endometrial cancer: an NRG oncology study. *Gynecologic Oncology: An International Journal*.

[3] Siebert M., Alyami M., Mercier F. (2021). Pressurized intraperitoneal aerosol chemotherapy (PIPAC) in association with systemic chemotherapy and bevacizumab, evaluation of safety and feasibility. A single center comparative study. *Surgical Oncology*.

[4] Ren T., Wang S., Shen Z. (2021). Efficacy and safety of bevacizumab plus oxaliplatin- or irinotecan-based doublet backbone chemotherapy as the first-line treatment of metastatic colorectal cancer: a systematic review and meta-analysis. *Drug safety: An international journal of medical toxicology and drug experience*.

[5] Halmos (2021). Pembrolizumab plus chemotherapy versus atezolizumab plus chemotherapy plus /& minus;bevacizumab for the first-line treatment of non-squamous NSCLC: a matching-adjusted indirect comparison. *Lung cancer: Journal of the International Association for the Study of Lung Cancer*.

[6] Chu G., Liu X., Yu W., Chen M., Dong L. (2021). Cisplatin plus paclitaxel chemotherapy with or without bevacizumab in postmenopausal women with previously untreated advanced cervical cancer: a retrospective study. *BMC Cancer*.

[7] Sabatier R., Pierga J. Y., Curé H. (2021). Circulating tumor cells and bevacizumab pharmacokinetics during neoadjuvant treatment combining chemotherapy and bevacizumab for early breast cancer: ancillary analysis of the AVASTEM trial. *Cancers*.

[8] Nissen N. I., Kehlet S., Boisen M. K. (2021). Prognostic value of blood-based fibrosis biomarkers in patients with metastatic colorectal cancer receiving chemotherapy and bevacizumab. *Scientific Reports*.

[9] Ayhan A., Akilli H. (2021). Prognostic factors associated with cytoreductive surgery plus hyperthermic intraperitoneal chemotherapy in recurrent ovarian cancer. *International journal of gynecology and obstetrics*.

[10] Lorusso D., Maltese G., Sabatucci I. (2021). Phase I study of rucaparib in combination with bevacizumab in ovarian cancer patients: maximum tolerated dose and pharmacokinetic profile. *Targeted Oncology*.

[11] Taira Y., Shimoji Y., Nakasone T. (2021). A case of nasal septal perforation caused by bevacizumab for advanced cervical cancer. *The journal of obstetrics and gynaecology research*.

[12] Pignata S., Lorusso D., Joly F. (2021). Carboplatin-based doublet plus bevacizumab beyond progression versus carboplatin-based doublet alone in patients with platinum-sensitive ovarian cancer: a randomised, phase 3 trial. *The Lancet Oncology*.

[13] García-Alfonso P., Díaz-Rubio E., Abad A. (2021). First-line biological agents plus chemotherapy in older patients with metastatic colorectal cancer: a retrospective pooled analysis. *Drugs and Aging*.

[14] Kanemitsu Y., Shitara K., Mizusawa J. (2021). Primary tumor resection plus chemotherapy versus chemotherapy alone for colorectal cancer patients with asymptomatic, synchronous unresectable metastases (JCOG1007; iPACS): a randomized clinical trial. *Journal of Clinical Oncology*.

[15] Tamiya M., Tamiya A., Suzuki H. (2021). Phase 2 study of bevacizumab plus carboplatin/nab-paclitaxel followed by bevacizumab plus nab-paclitaxel for non-squamous non-small cell lung cancer with malignant pleural effusion. *Investigational New Drugs*.

[16] Huang L. T., Cao R., Wang Y. R. (2021). Clinical option of pemetrexed-based versus paclitaxel-based first-line chemotherapeutic regimens in combination with bevacizumab for advanced non-squamous non-small-cell lung cancer and optimal maintenance therapy: evidence from a meta-analysis of randomized control trials. *BMC Cancer*.

[17] Liu L. H., Zhou G. F., Lv H., Wang Z. C., Rao S. X., Zeng M. S. (2021). Identifying response in colorectal liver metastases treated with bevacizumab: development of RECIST by combining contrast-enhanced and diffusion-weighted MRI. *European Radiology*.

[18] Guilloteau A., Abrahamowicz M., Boussari O. (2021). Impact of time-varying cumulative bevacizumab exposures on survival: re-analysis of data from randomized clinical trial in patients with metastatic colo-rectal cancer. *BMC Medical Research Methodology*.

[19] Markovic S. N., Suman V. J., Javed A. (2020). Sequencing ipilimumab immunotherapy before or after chemotherapy (nab-paclitaxel and bevacizumab) for the treatment of BRAFwt (BRAF wild-type) metastatic malignant melanoma. *American Journal of Clinical Oncology*.

[20] Miyashita M., Hattori M., Takano T., Toyama T., Iwata H. (2020). Risks and benefits of bevacizumab combined with chemotherapy for advanced or metastatic breast cancer: a meta-analysis of randomized controlled trials. *Breast cancer: the journal of the Japanese Breast Cancer Society*.

[21] Kim S. A., Kim J. W., Suh K. J. (2020). Conversion surgery after cetuximab or bevacizumab plus FOLFIRI chemotherapy in colorectal cancer patients with liver- and/or lung-limited metastases. *Journal of Cancer Research and Clinical Oncology*.

[22] Sadahiro S., Suzuki T., Okada K. (2020). Oral S-1 with 24-h infusion of irinotecan plus bevacizumab versus FOLFIRI plus bevacizumab as first-line chemotherapy for metastatic colorectal cancer: an open-label randomized phase II trial. *Oncology*.

[23] Catalano V., Bergamo F., Cremolini C. (2020). Clinical impact of first-line bevacizumab plus chemotherapy in metastatic colorectal cancer of mucinous histology: a multicenter, retrospective analysis on 685 patients. *Journal of Cancer Research and Clinical Oncology*.

[24] Ferrari A., Merks J. H., Chisholm J. C. (2020). Outcomes of metastatic non-rhabdomyosarcoma soft tissue sarcomas (NRSTS) treated within the BERNIE study: a randomised, phase II study evaluating the addition of bevacizumab to chemotherapy. *European journal of cancer*.

[25] Gunjur A., Chong G., Lim A. (2020). Occult gastrointestinal perforation in a patient with EGFR-mutant non-small-cell lung cancer receiving combination chemotherapy with atezolizumab and bevacizumab: Brief Report. *Clinical lung cancer*.

